# Prostate Cancer Cell Lines under Hypoxia Exhibit Greater Stem-Like Properties

**DOI:** 10.1371/journal.pone.0029170

**Published:** 2011-12-28

**Authors:** Yuanyuan Ma, Dongming Liang, Jian Liu, Karol Axcrona, Gunnar Kvalheim, Trond Stokke, Jahn M. Nesland, Zhenhe Suo

**Affiliations:** 1 Department of Pathology, University of Oslo, The Norwegian Radium Hospital, Oslo University Hospital, Oslo, Norway; 2 Department of Urology, University of Oslo, The Norwegian Radium Hospital, Oslo University Hospital, Oslo, Norway; 3 Department of Cell Therapy, University of Oslo, The Norwegian Radium Hospital, Oslo University Hospital, Oslo, Norway; 4 Department of Radiation Biology, Institute for Cancer Research, University of Oslo, The Norwegian Radium Hospital, Oslo University Hospital, Oslo, Norway; 5 Department of Pathology, Faculty of Medicine, Institute of Clinical Medicine, University of Oslo, Oslo, Norway; The University of Texas M.D Anderson Cancer Center, United States of America

## Abstract

Hypoxia is an important environmental change in many cancers. Hypoxic niches can be occupied by cancer stem/progenitor-like cells that are associated with tumor progression and resistance to radiotherapy and chemotherapy. However, it has not yet been fully elucidated how hypoxia influences the stem-like properties of prostate cancer cells. In this report, we investigated the effects of hypoxia on human prostate cancer cell lines, PC-3 and DU145. In comparison to normoxia (20% O_2_), 7% O_2_ induced higher expressions of HIF-1α and HIF-2α, which were associated with upregulation of Oct3/4 and Nanog; 1% O_2_ induced even greater levels of these factors. The upregulated *NANOG* mRNA expression in hypoxia was confirmed to be predominantly retrogene *NANOGP8*. Similar growth rates were observed for cells cultivated under hypoxic and normoxic conditions for 48 hours; however, the colony formation assay revealed that 48 hours of hypoxic pretreatment resulted in the formation of more colonies. Treatment with 1% O_2_ also extended the G_0_/G_1_ stage, resulting in more side population cells, and induced CD44 and ABCG2 expressions. Hypoxia also increased the number of cells positive for ABCG2 expression, which were predominantly found to be CD44^bright^ cells. Correspondingly, the sorted CD44^bright^ cells expressed higher levels of ABCG2, Oct3/4, and Nanog than CD44^dim^ cells, and hypoxic pretreatment significantly increased the expressions of these factors. CD44^bright^ cells under normoxia formed significantly more colonies and spheres compared with the CD44^dim^ cells, and hypoxic pretreatment even increased this effect. Our data indicate that prostate cancer cells under hypoxia possess greater stem-like properties.

## Introduction

Somatic tumors, including prostate cancer, contain a small subset of stem-like cells, called cancer stem cells, with capacities for self-renewal, differentiation, and initiation of new tumors. It has been demonstrated that cancer stem cells can escape from radiotherapy and chemotherapy, and are able to form metastatic tumors in other organs [1], [2]. Cancer stem cells preferentially reside in specific hypoxic microenvironment-niches, often existing inside tumors [3], [4].

The hypoxia inducible factors (HIFs) are key regulators found in mammalian cells under lower oxygen tension; they are involved with multiple functions, such as cell survival, angiogenesis, and stem cell maintenance, and play essential roles in cellular and systemic homeostasis in response to hypoxia [5]. HIFs are heterodimers; *HIF1A* (HIF-1α) and *EPAS1* (HIF-2α) are the two major isoforms of the α-subunit, and share a high degree of sequence homology. Oct3/4 (also called POU5F1) and Nanog are embryonic stem cell markers that are important for transcription and in maintaining self-renewal of embryonic stem cells and primordial germ cells. They have also been identified in different somatic tumors, including head and neck, lung, colorectal, ovarian, and prostate cancers [6]–[11]. Comparatively, the expressions of these genes are down-regulated in all differentiated somatic cell types, *in vitro* as well as *in vivo* [12], [13]. *NANOG*, also called *NANOG1*, has several pseudogenes, and among them *NANOGP8* has later been confirmed to be a retrogene. Both *NANOG1* and *NANOGP8* expressions have been identified in different cancer cell types [14], [15], including prostate cancer cells [16].

A number of surface markers have been used to isolate putative cancer stem/progenitor cells. In prostate cancer, the early progenitor cells are associated with several specific surface markers, such as CD44, CD133, and CXCR4 [17]–[19]. Side population technology has also been used to isolate cancer stem cells with the ability to pump out Hoechst 33342 [20]. Efflux of the dye is attributed to members of the ATP-binding cassette family, such as ABCG2 (breast cancer resistance protein, BCRP). The upregulation of ABCG2 is also responsible for chemotherapeutic resistance in certain cancer cells [21]. In breast and prostate cancers, previous studies have identified CD44^+^ or CD117^+^/ABCG2^+^ cells with stem-like characteristics, such as increased clonogenic/tumorigenic properties, higher expressions of stemness genes, and stronger ability to form tumors in animal models [19], [22], [23].

Hypoxia helps embryonic stem cells to maintain stemness and higher oxygen tensions drive cells into proliferation and differentiation, which are more susceptible to conventional treatment modalities [24], [25]. Similar results have been observed in adult cells, like adipocytes, fibroblasts, and several types of cancer cells [26]–[28]. However, the effects of hypoxia on prostate cancer cells have not been fully elucidated. Therefore, in this study we examined the prostate cancer cell lines PC-3 and DU145 at different oxygen tensions in order to better understand the effect of hypoxia on the stem-like properties of the cells. Stemness factors, Oct3/4 and Nanog, were expressed at higher levels in the cells under hypoxic cultivation and these cells exhibited elevated colony formation potential compared to the cells under normoxic condition. Furthermore, the upregulated *NANOG* mRNA expression under hypoxia was confirmed mainly derived from the retrogene *NANOGP8*. In these prostate cancer cell lines, hypoxia also increased the fraction of side population cells, extended the G_0_/G_1_ stage and resulted in higher levels ABCG2 and CD44 expressions. Additional experiments demonstrated that CD44^bright^ cells exhibited significantly greater stemness, as verified by colony formation assay, sphere growth assay, and stemness factor expression analyses.

## Materials and Methods

### Cell culture

Human prostate cancer cell lines, PC-3 and DU145, were purchased from ATCC (American Type Culture Collection, USA) and maintained in our lab for this study. For conventional cell culture, cells were seeded in culture flasks with RPMI 1640 medium supplemented with 10% fetal bovine serum, 100 units/ml penicillin, and 100 µg/ml streptomycin. Cultures were maintained at 37°C in a humidified incubator in an atmosphere of 20% O_2_, 5% CO_2_, and 75% N_2_.

The Xvivo Closed Incubation System (Xvivo system 300 C, BioSpherix, New York, USA) was used in this study in order to accurately maintain different oxygen tensions in different chambers. After 24 hours of cultivation in conventional cell culture (allowing cells to attach onto the flasks), the cells were transferred into different chambers with 1% O_2_, 5% CO_2_, and 94% N_2_; 7% O_2_, 5% CO_2_, and 88% N_2_; or 20% O_2_, 5% CO_2_ and 75% N_2_ for variable periods of time before being harvested for additional analysis.

### Semiquantitative reverse transcription-PCR (RT-PCR)

Total RNA was extracted from the cultivated cells using the RNeasy Kit (Qiagen, CA, USA) according to the manufacturer's instruction. To eliminate any DNA, DNase I was used in the RNA isolation procedure. RNA sample concentrations were quantified using a spectrophotometer (Nanodrop ND-1000, USA) at OD260/280.

Complementary DNA (cDNA) was subsequently synthesized from 5 µg total RNA using the Multiscribe reverse transcriptase (Applied Biosystems, Foster City, CA). The conditions for reverse transcription were: 25°C for 10 minutes, 37°C for 12 minutes, 85°C for 5 minutes, followed by holding at 4°C. cDNA was stored at −70°C for later PCR analyses.

PCR amplification of cDNA was performed using a PCR system (DOPPIO VWR, UK) and the following program: initial denaturation at 95°C for 10 minutes; followed by 30 cycles (28 cycles for GAPDH) of annealing at 60°C for 30 seconds, and extension at 72°C for 30 seconds; followed by termination with a 10 minute elongation step at 72°C. The primers used for RT-PCR were: for Nanog, F 5′-ATGCCTCACACGGAGACTGT-3′ and R 5′-AGGGCTGTCCTGAATAAGCA-3′, amplifying a 66-bp fragment; for Oct3/4, F 5′-ACATGTGTAAGCTGCGGCC-3′ and R 5′-GTTGTGCATAGTCGCTGCTTG-3′, amplifying a 297-bp fragment; for HIF-1α, F 5′-AGTGTACCCTAACTAGCCGAGGAA-3′ and R 5′-CTGAGGTTGGTTACTGTTGGTATCA-3′, amplifying a 113-bp fragment; for HIF-2α, F 5′-GACCAGCAGATGGACAACTTGTAC-3′ and R 5′-CAGAAAGATCATGTCGCCATCTT-3′, amplifying a 84-bp fragment; and for GAPDH, F 5′-CCTCAAGATCATCAGCAATGC-3′ and R 5′-TGGTCATGAGTCCTTCCACG-3′, amplifying a 101-bp product. The experiments were repeated at least three times.

The amplified PCR products were separated by 7.5% polyacrylamide gel electrophoresis, stained with GelRed (Molecular Probes, Invitrogen), and visualized with a syngene image system (G: BOX Syngene, USA).

The mRNA expressions of *NANOG1* and *NANOGP8* were measured by quantitative PCR using a Taqman ABI 7900 Sequence Detector System (Applied Biosystems). The published specific primers and probes [29] were used in this study . For *NANOG1*: forward primer was 5′-CGCCCTGCCTAGAAAAGACATTT -3′, reverse primer was 5′-AGAAGCCGTCTCTGGCTATAGATAA -3′, and the probe was CTGCTAAGGACAACATTGAT; for *NANOGP8*: forward primer was 5′-CGCCCTGCCTAGAAAAGACATTT-3′ , reverse primer was 5′-ACGAGTTTGGATATCTTTAGGGTTTAGAATC-3′, and the probe was CCTTGGCTGCCGTCTCTG. All the primers and probes labeled with FAM-MGB were obtained from Applied Biosystems. The GAPDH was used as an internal control and the Ct values at 20% O_2_ were used as calibrators for evaluating *NANOG1* and *NANOGP8* expression levels in response to hypoxia. The experiments were performed in duplicate. The expression levels of the *NANOG1* and *NANOGP8* were analyzed through the ΔΔCt method [29].

### Immunoblotting

Cells were quickly rinsed with ice-cold phosphate-buffered saline (PBS) and scraped into RIPA buffer (25 mM Tris HCl pH 7.6, 100 mM NaCl, 1% NP40, 1% sodium deoxycholate, 0.1% SDS; Thermo Scientific Pierce, Germany), with protease inhibitors (0.1 µM aprotinin, 1.0 mM PMSF, 1 µM leupeptin, 1 µM pepstatin) added immediately before use. The samples were centrifuged at 15,000 rpm for 15 minutes at 4°C and the supernatants were transferred to new tubes. The protein concentrations were measured with a Bio-Rad protein assay according to the manufacturer's instruction. The samples were heated with a benchtop heater (Model 111002, Boekel Scientific, USA) at 100°C for 5 minutes in SDS-loading buffer (500 mM Tris-HCl pH 6.8; 10% Glycerol, 2% SDS, 0.6 M DTT, 0.05% bromophenol blue), and then an equal amount of protein (50 µg) per sample was subjected to 10% SDS-PAGE and transferred to polyvinylidene difluoride transfer membrane (BIO-RAD, USA). Membranes were blocked with 5% non-fat dry milk in TBS-Tween for 60 minutes at room temperature and then incubated with the primary antibodies at optimal dilution in TBST/5% milk overnight at 4°C. The optimized antibodies used in this study included: HIF-1α (1 µg/ml MAB1536, R&D), HIF-2α (1 µg/ml MAB2886, R&D), GAPDH (0.2 µg/ml AF5718, R&D), Oct3/4 (1 µg/ml MAB1759, R&D), Nanog (1 µg/ml AF1997, R&D), and ABCG2 (0.5 µg/ml B7059, Sigma-Aldrich). The membranes were then incubated with secondary HRP-conjugated antibodies and immunocomplexes were visualized by enhanced chemiluminescence (GE Healthcare, UK). Western blotting experiments were repeated at least three times.

### Cell block preparation

Cells were grown to 80% confluence and then were digested with 0.25% trypsin and EDTA (Invitrogen, USA), harvested, and centrifuged at 2000 rpm for 10 minutes. Supernatants were discarded, 3 drops of plasma and 2 drops of thrombin were added to the sedimentation, and the contents were carefully mixed by tube rotation. One minute later, the mixture was coagulated and 4% buffered formalin was added to the tube for fixation. The coagulated mass was then placed in linen paper and used to construct a paraffin block by the conventional process.

### Immunocytochemistry

Cell blocks were sliced into 4-µm paraffin sections that were then deparaffinized using PT-Link apparatus. Next, the sections were rinsed with DAKO wash buffer, incubated with hydrogen peroxide for 5 minutes, and then incubated with primary antibody for 30 minutes at room temperature. The antibodies used and their concentrations were: HIF-1α (mouse, 1∶200; catalog number: NB100-150, Novus), HIF-2α (rabbit, 1∶100; catalog number: NB100-122, Novus), Oct3/4, (goat, 10 µg/ml; catalog number: AF1759, R&D) and Nanog (goat, 5 µg/ml; catalog number: AF1997, R&D).

After another rinse with DAKO wash buffer, mouse/rabbit EnVision FLEX+Linker reagent was added and samples were incubated for 15 minutes at room temperature, followed by incubation with EnVision FLEX+HRP for 30 minutes at room temperature. Samples with primary antibodies from goat were incubated for 30 minutes at room temperature with mouse anti-goat IgG before the addition of mouse EnVision FLEX+Linker reagent and EnVision FLEX+HRP as described above. The sections were rinsed, color reaction developed with DAB reagent, counterstained in hematoxylin for 20 seconds, dehydrated, and mounted under glass cover slips in preparation for evaluation by microscopy.

### Cell counting (cell proliferation rate)

Cell proliferation was evaluated by counting cell numbers using the Electronics Countess Automated Cell Counter (Invitrogen, USA). After trypsinization, the floating cells were collected to create a cell suspension that contained no obvious cell clusters. In each preparation, 10 µl of cell suspension was mixed with 0.4% trypan blue dye (1∶1) before being loaded onto a cell counting chamber slide for cell counting. The number of viable cells that were able to exclude the dye was counted for each experimental condition. For each sample, the cell number was counted at least three times.

### Colony formation assay

Using six-well plates, 500 cells per well were maintained in oxygen tensions of 1%, 7%, and 20% for 48 hours. All plates were then placed in an incubator with 20% O_2_ for 2 weeks for observation of colony formation. Colonies were fixed with 4% buffered formalin for 15 minutes, and then stained with 1% crystal violet for 30 minutes. The plates were gently washed with PBS and dried before microscopic colony evaluation. Colonies that contained more than 30 cells were counted. Colony formation efficiency was calculated as follows: colony formation efficiency = colonies/input cells×100%. Data are representative of three independent experiments.

### Cell cycle analysis

After incubation under different oxygen tensions, including 1% or 20% O_2_, the PC-3 and DU145 cells were harvested and fixed with methanol at −20°C overnight. These cells were used to prepare a single cell suspension to which was added 1.5 µg/ml of Hoechst 33258 before the cells were kept on ice for 30 minutes. After that, the samples were analyzed with an LSRII flow cytometer (Becton Dickinson, San Jose, CA, USA).

### Side population assay

Cells grown to 80% confluence (about 1×10^6^ cells) were harvested and suspended in prewarmed RPMI 1640 medium containing 2% fetal bovine serum and 2 mM HEPES buffer. Hoechst 33342 dye (stock solution of 1 mg/ml; Sigma) was then added to a final concentration of 5 µg/ml, and the mixture was incubated with intermittent shaking for 90 minutes at 37°C, in the presence or absence of verapamil (50 µM; Sigma). Then, the cells were washed with ice-cold HBSS with 2% FBS, centrifuged at 4°C, and resuspended in ice-cold HBSS containing 2% FBS. Propidium iodide was added to the suspended cells to a final concentration of 2 µg/ml, in order to reveal viable cells. Before analysis, the cells were filtered through a 70-µm cell strainer to obtain a single cell suspension. The cell aggregates were discarded from the analysis by doublet discrimination and single cells were analyzed on a LSRII flow cytometer (BD Biosciences). Hoechst 33342 dye was excited at 350 nm and the side-population cells were visualized by the use of red (red, 660/10 nm) vs. blue (blue, 424/44 nm) detection.

### ABCG2/CD44 phenotype and Fluorescence-activated cell sorting (FACS)

After 48 hours of incubation at oxygen tensions of 1% and 20%, the PC-3 and DU145 cells were trypsinized, counted, washed with cold FACS buffer (PBS+BSA 0.03%), and resuspended to a final concentration of 10^6^ cells/ml. The cells were pre-blocked with 5% BSA for 30 minutes on ice before they were stained with primary antibodies (anti-CD44 monoclonal antibody directly conjugated with APC (allophycoyanin) and anti-ABCG2 monoclonal antibody directly conjugated with FE (phycoerythin); BD Pharmingen Company) on ice, in the dark, for 30 minutes. Cell suspensions were washed twice, resuspended in 400 µl FACS buffer, and filtered through a 70-µm nylon mesh. Samples were analyzed on a flow cytometer (Becton Dickinson, San Jose, CA, USA) for detection of ABCG2 and CD44, and a FACS DiVa cell sorter was used for cell sorting. After cultivation at 1% or 20% O_2_ for 48 hours, the PC-3 and DU145 cells were sorted based on CD44 expression. For the CD44 positive cells, only the top 10% expressing cells were selected (called CD44^bright^); for the CD44 negative cells, the bottom 10% expressing cells were isolated (called CD44^dim^). For each sample, viable and single cells were gated; APC Mouse IgG2b (BD Pharmingen, USA) and FE Mouse IgG2b (BD Pharmingen, USA) isotype controls were used as negative controls.

### Sphere formation assay

The assay used was based on previously described methods [30]. After the CD44^bright^ cells were sorted with the method as described above, single CD44^bright^ and CD44^dim^ cells were plated at a density of 300 cells per well, in ultralow attachment six-well plates (Ultra low cluster plates, Life sciences). These cells were cultivated in serum free DMEM/F12 medium (Invitrogen) supplemented with 20 ng/ml EGF and 20 ng/ml bFGF for ten days under normoxia conditions before the spheres were evaluated under inverse miscopy and counted (more than 30 cells within a sphere was considered to be a full sphere). Data are representative of three independent experiments.

### Statistical analyses

For each experiment, data are shown as mean ± SEM of at least three independent experiments; SPSS software (version 16.0) was used for data analysis. Statistical analyses were performed using the one-way ANOVA test and Student's *t*-test (*P*<0.05 was considered statistical significance).

## Results

### Hypoxia induces expression of HIF-1α, HIF-2α, Oct3/4 and Nanog

HIF-1α and HIF-2α, the major transcriptional factors responding to hypoxia, were examined in human prostate cancer cells PC-3 and DU145 that were exposed to different oxygen tensions for variable periods of time. At 20% O_2_ tension, HIF-1α and HIF-2α were weakly expressed at both the mRNA and protein levels; comparatively higher levels of HIF-1α and HIF-2α expression were observed at 7% O_2_ tension, and the highest levels were seen at 1% O_2_ tension (Figure 1A). At reduced oxygen tension levels, these two factors were already upregulated after 6 hours of cultivation. Their expressions reached the highest levels at 12 hours of cultivation at 7% O_2_ tension, but reached highest levels at only 6 hours of cultivation at 1% O_2_. Protein expression after 48 hours of cultivation at different oxygen tensions was also studied by immunocytochemistry (Figure 1B). The expressions of HIF-1α and HIF-2α were consistently higher in the hypoxia-treated cells, in agreement with the findings obtained by RT-PCR and immunoblotting.

**Figure 1:** Hypoxia increases the expressions of HIF-1α and HIF-2α. (A) In comparison to the cells cultivated at 20% O_2_, the cells cultivated at 7% O_2_ show higher levels of HIF-1α and HIF-2α, and the cells cultivated at 1% O_2_ show the highest levels of HIF-1α and HIF-2α by both RT-PCR and immunoblotting. (B) Immunocytochemistry reveals higher levels of HIF-1α and HIF-2α expressions in the cells cultivated under 7% O_2_ and the highest levels of HIF-1α and HIF-2α expressions in the cells cultivated under 1% O_2_ for both cell lines. The breast carcinoma sections were used as positive controls for both HIF-1α and HIF-2α. All photos were originally taken at 200× and all the insets were taken at 400×.

Oct3/4 and Nanog are frequently used as markers for the undifferentiated cells and play an essential role in sustaining capacity of self-renewal in adult stem cells [31], [32]. The expressions of these transcription factors were also examined in PC-3 and DU145 cells that were cultivated at different oxygen tensions. At both the mRNA and protein levels (Figure 2A), weak expressions of Oct3/4 and Nanog were revealed in these two cell lines cultivated at 20% O_2_ tension, while their expressions were upregulated in cells cultivated under 7% and 1% O_2_ conditions. In both cell lines, the expressions of these two factors were higher at 1% O_2_ than at 7% O_2_. As was also seen in immunoblotting analyses (Figure 2A), Oct3/4 and Nanog began to substantially increase as early as 6 hours after the cells were transferred to 1% O_2_, and reached maximum levels at 12 hours for both cell lines. When the cells were placed in 7% O_2_, the expressions of these two factors were also substantially elevated after 6 hours, and reached the highest levels at 12 hours cultivation; however, these expression levels were weaker than those observed in cells exposed to 1% O_2_. Similar results were also obtained by immunocytochemistry (Figure 2B). Following exposure to hypoxic condition, enhanced Oct3/4 and Nanog expressions were seen in both PC-3 and DU145 cells.

**Figure 2:** Hypoxia increases the expressions of Oct3/4 and Nanog. (A) In comparison to the cells cultivated at 20% O_2_, the cells cultivated at 7% O_2_ show higher levels of Oct3/4 and Nanog expressions, and the cells cultivated at 1% O_2_ show the highest levels of Oct3/4 and Nanog expressions in PC-3 and DU145 cell lines by both RT-PCR and immunoblotting. (B) Immunocytochemistry reveals corresponding higher levels of Oct3/4 and Nanog expressions at 7% O_2_ and the highest levels of Oct3/4 and Nanog expressions at 1% O_2_, in comparison to the cells cultivated at 20% O_2_ for both cell lines. Human seminoma tissue sections were used as positive controls for these two antibodies. All photos were originally taken at 200× and all the insets were taken at 400×.

To determine whether the elevated *NANOG* expression was derived from *NANOG1* or *NANOGP8*, quantitative RT-PCR analyses were further performed, with the corresponding cells cultivated under normoxia as calibrators. It was repeatedly verified that the *NANOG1* expression in the cells under normoxia was at very low level, with average Ct values 37.24 and 37.37 for the PC-3 cell and DU145 cells, respectively. However, the *NANOGP8* expression in the cells under normoxia was relatively high, with average Ct values 33.56 and 33.51 for the PC-3 cell and DU145 cells, respectively. Although higher levels *NANOG1* and *NANOGP8* expressions could be observed in both cell lines under hypoxia, the elevated *NANOG* expression was confirmed predominantly *NANOGP8*, with up to 6-fold and 10-fold increase in expression in the PC-3 and DU145 cells under 1% O_2_, respectively (Figure 3). Since the *NANOG1* expression in the cells under normoxia was extremely low, the 2.6-fold and 3.1-fold increase in expression of this gene in the PC-3 and DU145 cells under 1% O_2_ represented still quite low expression level.

**Figure 3:** Quantitative PCR results of *NANOG1* and *NONOGP8*. Compared to the cells under normoxia, there are elevated *NANOG1* and *NONOGP8* expressions in the cells under 7% O_2_ for both cell lines, with up to 1.8-fold increase *NANOG1* expression and up to 2.5-fold *NONOGP8* increase in both cell lines; the cells under 1% O_2_ express even higher levels of *NANOG1* and *NONOGP8*, with 2.6-fold and 3.1-fold increase in *NANOG1* expression in the PC-3 and DU145 cell lines, respectively, and with 6-fold and 10-fold increase in *NONOGP8* expressions in the PC-3 and DU145 cell lines, respectively.

### Hypoxia increases colony formation capability and extends G_0_/G_1_ stage

Since hypoxia increased the expression of stemness factors, we next investigated whether hypoxia influenced the proliferation of these cells. The PC-3 and DU145 cells were cultivated under normoxia (20% O_2_) or hypoxia conditions (1% O_2_ and 7% O_2_) for 48 hours for the proliferation assay. As shown in Figure 4A, for each cell line there were no statistically significant differences in proliferation of the cells cultivated at different oxygen tensions (*P*>0.05), although the cells grew somewhat slower under hypoxia than normoxia. Next, we asked whether hypoxia-pretreatment could influence clonogenicty in these cells. The cells were initially exposed to different oxygen tensions for 48 hours, followed by transfer to a normoxic chamber (20% O_2_) for 14 days for the colony formation assay. Compared to the cells that were steadily cultivated at 20% O_2_, more colonies were observed in the cells that were pretreated at 7% O_2_, and even more colonies were seen in the cells pretreated at 1% O_2_ (Figure 4B). Compared to the cells always cultivated under normoxia, statistically significantly higher colony formation efficiency was identified in the hypoxia-pretreated PC-3 and DU145 ells (Figure 4C). Cell cycle analyses demonstrated an extended G_0_/G_1_ stage in the cells that were exposed to 1% O_2_ for 48 hours in comparison with the cells cultivated at 20% O_2_ as controls (*P*<0.05) (Figure 4D and E), indicating more cells in a quiescent status under hypoxia.

**Figure 4:** Hypoxic effects on cell proliferation, colony formation and cell cycle. (A) Cell proliferation curves show no statistical difference for cell growth under different oxygen tensions (*P>0.05*). (B) Colony formation assay for both cell lines shows more colonies in the cells pre-treated at 7% O_2_ for 48 hours and even more colonies in the cells pre-treated under 1% O_2_ (C) Histograms for the colony formation efficiency shows statistically higher efficiency in the cells pre-treated under hypoxia (7% or 1% O_2_) for both cell lines (*P*<0.0001). (D) Flow cytometry shows extended G_0_/G_1_ stage for both cell lines which have been cultivated under 1% O_2_ for 48 hours, in comparison to the cells always kept under normoxia. (E) Statistical analyses reveal significantly extended G_0_/G_1_ stage in the cells cultivated under hypoxia for both cell lines (*P*<0.05).

### Hypoxia increases the fraction of cells with stem-like phenotype

Side population cells, assumed to contain putative prostate cancer stem cells, are known to pump out the dye Hoechst 33342 [20], [33]. Cells exhibiting this activity were further assessed during cultivation at different oxygen tensions. Higher fractions of these side population cells were observed in cultures kept at 1% O_2_ tension for 48 hours in comparison to the cells cultivated at 20% O_2_ (Figure 5A and B).

**Figure 5:** Stem-like phenotype analyses by flow cytometry. PC-3 and DU145 cells were cultivated in 1% O_2_ and 20% O_2_ coditions for 48 hours to analyze stem-like phenotype through flow cytometry assay. (A) The representative images show that side population cells were induced in both cell lines after hypoxic treatment. (B) Statistic analyses show significant difference in side population. (C) Flow cytometry analyses show higher levels of ABCG2 expression intensity in both cell lines under hypoxia. (D) Histogram shows statistically significant difference in ABCG2 expression. (E) Flow cytometry analyses show higher CD44 expression intensity in both cell lines under hypoxia. (F) Histogram shows statistically significant difference in CD44 expression.

ABCG2 and CD44 have been described as prostate cancer stem-like markers based on clinical investigations and studies in prostate cancer cell lines [19], [33]. Therefore, ABCG2 and CD44 expressions in the PC-3 and DU145 cells that were incubated at 1% or 20% O_2_ tensions for 48 hours were examined with flow cytometry. As shown in Figures 5C and D, threw were 1.20-fold and 1.42-fold increase in ABCG2 expression in the PC-3 and DU145 cells under 1% O_2_, respectively, in comparison to the cells always cultivated under normoxia. Similarly, there were 1.50-fold and 1.45-fold increases in CD44 expression in the PC-3 and DU145 cells under 1% O_2_, respectively, in comparison to the cells always cultivated under normoxia (Figures 5E and F).

Since hypoxia could induce both ABCG2 and CD44 expression in both cell lines, we further investigated the relationship between CD44 and ABCG2. Double staining of these two surface markers revealed that the hypoxia-induced ABCG2^+^ cells were primarily CD44^bright^ cells, and the CD44^dim^ cells under the same culture condition were mostly negative for ABCG2 expression (Figure 6A).

**Figure 6:** CD44^bright^ cells are mainly positive for ABCG2, Oct3/4 and Nanog. (A) Double staining of CD44 and ABCG2 surface markers with flow cytometry assay shows higher levels expressions of these factors in both cell lines under hypoxia for 48 hours. (B) The CD44^bright^ cells under normoxia express higher levels of ABCG2, Oct3/4 and Nanog, but the CD44^dim^ cells under the same normoxia condition express very low levels of these factors. The CD44^bright^ cells pretreated under 1% O_2_ for 48 hours show even higher levels of these factors compared to the CD44^bright^ cells cultivated under normoxia.

### CD44^bright^ cells show stem-like properties

The sorted CD44^bright^ and CD44^dim^ cells were further examined by immunoblotting. As shown in Figure 6B, in both PC-3 and DU145 cell lines grown under normoxia, the CD44^bright^ cells expressed higher levels of ABCG2, Oct3/4, and Nanog than the CD44^dim^ cells. Hypoxic pretreatment of these cell lines for 48 hours resulted in even greater levels of expression of these factors in the CD44^bright^ cells.

After verifying the higher stemness factor and ABCG2 expressions in the CD44^bright^ cells, both under hypoxia and normoxia, we examined whether the CD44^bright^ cells had greater colony formation capability (a property of stem-like cells). As can be seen in Figures 7A and 7B, the CD44^bright^ cells formed significantly more colonies compared to the CD44^dim^ cells. Next, we tested how the CD44^bright^ and CD44^dim^ cells responded to hypoxic pretreatment (1% O_2_), in comparison to the cells consistently cultivated at normoxia. The CD44^bright^ cells which were hypoxic-pretreated for 48 hours could form significantly more colonies than the CD44^bright^ cells without hypoxic pretreatment.

**Figure 7:** CD44^bright^ cells show stem-like properties. (A) For both PC-3 and DU145 cell lines, more colonies are shown in the CD44^bright^ cells than the CD44^dim^ cells under nomoxia condition, while even more colonies can be seen in the CD44^bright^ cells pretreated under 1% O_2_ for 48 hours. (B) Histograms for the colony formation efficiency show statistically significantly higher efficiency in the CD44^bright^ cells than the corresponding CD44^dim^ cells (*P*<0.0001 for both cell lines), and even higher level efficiency in the hypoxia- pretreated CD44^bright^ cells in comparisons with the CD44^bright^ cells without hypoxic pretreatment (*P*<0.05 for both cell lines). (C) Sphere formation assay shows spheres in the CD44^bright^ cells in both normoxia and hypoxic pretreated cells while there is no qualified sphere in the corresponding CD44^dim^ cells for both cell lines. (D) Histograms show sphere formation efficiency in the CD44^bright^ and CD44^dim^ cells with and without hypoxia pretreatment.

The sorted subpopulations of CD44^bright^ and CD44^dim^ cells were additionally examined by sphere growth assays since sphere growth is common in stem-like cells. As shown in Figure 7C, the CD44^dim^ cells hardly formed any sphere, no matter the cells were hypoxia pre-treated or not. However, there was a great number of spheres in the CD44^bright^ cells from both cell lines, either from the nomoxia or from the hypoxia pretreatment. Although there was no significant sphere formation efficiency difference in the hypoxia pre-treated CD44^bright^ cells compared to the nomoxia pre-treated CD44^bright^ cells in both cell lines, the hypoxia pre-treated CD44^bright^ cells in the PC-3 cell line demonstrated a 1.21-fold increase in sphere formation efficiency, and the hypoxia pre-treated CD44^bright^ cells in the DU145 cells revealed a 1.14-fold increase in sphere formation efficiency, in comparison with their control cells.

## Discussion

Hypoxia often occurs in the inner part of solid tumors, creating an environment where undifferentiated tumor cells can exist. For prostate cancer, hypoxia is commonly associated with poor prognosis [34]. In this study, we have demonstrated that hypoxia can upregulate stem-like properties of the prostate cancer cell lines PC-3 and DU145. It has been hypothesized that cancer stem-like cells may persist as a distinct population within tumors and cause relapse and metastasis following general cancer therapies like radiotherapy and chemotherapy. Therefore, it is of great value to identify factors that affect the stem-like properties of cancer cells and to determine what conditions influence the differentiation of stem cells.

The hypoxia inducible factors HIF-1α and HIF-2α are reportedly activated in aggressive tumor cells [35], [36]. HIF-1α expression is increased in primary prostate cancers, prostate cancer bone marrow metastasis of PC-3 and brain metastasis of DU145, compared to in normal prostate epithelium [37], [38]. In this study, HIF-1α was weakly expressed under normoxia and their expressions were increased under hypoxic conditions. This is in agreement with earlier reports of higher expressions in response to hypoxia [39]–[41]. In our study, HIF-2α was also upregulated in response to hypoxia treatment in consistent with increased expression of HIF-1α. Moreover, in a clinical observation, HIF-1α expression was elevated in high-grade prostatic intraepithelial neoplastic lesions (the precursor of a majority of invasive prostate adenocarcinoma), relative to expression levels in normal epithelium, stromal cells, and benign prostatic hyperplasia [42].

The biological impact of hypoxia is exerted through transcriptional factors, such as Oct3/4 and Nanog [43]. Oct3/4 and Nanog are key players in a transcriptional network for maintenance of embryonic stem cell and primordial germ cells self-renewal [6], [11]. Our present study revealed that Oct3/4 and Nanog were expressed in the prostate cancer cell lines PC-3 and DU145, albeit in a lower level. Invasive tumor cells are shown with a stem-like genomic signature expressing a number of stem cell genes, including Oct3/4 and Nanog and these cells are more tumorigenic compared to their non-invasive counterpart [44]. In our present study, we found that the expressions of these genes were upregulated upon hypoxia exposure, at both the mRNA and protein levels, in parallel with the increasing expressions of HIF-1α and HIF-2α. The upregulation of Oct3/4 expression could be correlated with the enhanced HIF-2α expression under hypoxia and this observation is consistent with previous findings that HIF-2α binds to the promoter of Oct3/4 and induces its expression and activity directly [45], supporting a potential role for the interaction of HIF-2α and Oct3/4 in prostate cancer cells response to hypoxia.

In order to discriminate whether the upregulated *NANOG* mRNA expression was derived from *NANOG1* and/or *NANOGP8* genes in response to hypoxia, specific primers and probes were used to detect the expressions of these two genes in PC-3 and DU145 cell lines under different oxygen tensions by quantitative RT-PCR. In line with previous reports, there was extremely low level *NANOG1* expression in these cells [16], [29]. Although hypoxia could upregulate the expression of this gene in both cell lines, the expressions of the gene in these cells were still very low even in the cells under hypoxia. However, the *NANOGP8* was expressed in higher levels in both cell lines under normoxia, and its expression was greatly upregulated by hypoxia, with up to 6-fold and 10-fold increase in the PC-3 and DU145 cell lines, respectively, indicating that *NANOGP8* expression was predominantly influenced by hypoxia. Since Nanog protein expression was upregulated under hypoxia, and the cells under hypoxia revealed greater stem-like features, our results may support the notion that *NANOGP8* plays an important role on the cancer stem-like properties in prostate cancer cells [16], [29].

It is well documented that oxygen plays an important role in the development of tissues and cells. Hypoxia often occurs in pathophysiological conditions, especially when growth exceeds the blood supply in the tumor. It has been speculated that the formation of a hypoxic niche may drive selection of cancer stem cells that can maintain tumors by regulating specific developmental programs. Based on these reports, we wanted to know whether hypoxia influenced cell proliferation. Although there was no statistically significant difference between cells' proliferation under hypoxia compared to that under normoxia, the cells grew slowly under hypoxia with extended G0/G1, indicating higher quiescent status of these cells in hypoxia.

To study the effect of hypoxia on stem-like cell phenotypes, we assessed the fraction of side population cells. The side population assay has been successfully used for identification of cancer stem-like cells in studies of common urological malignancies, including prostate, bladder, and renal cancers [47]. Our experiments revealed a significantly higher number of side population cells in both the PC-3 and DU145 cells that were treated with 48 hours in 1% O_2_, strongly indicating that stem-like properties of these cancer cells could be greatly upregulate *in vitro*. Side population cells contain active ATP-cassette family members (e.g., ABCG2) that can pump Hoechst 33342 dye out of the cells and ABCG2 is associated with multi-drug resistance. Importantly, ABCG2 is a key molecular determinant for the side population cells and has been reviewed as a universal stem cell marker [33]. Consistent with the elevated fraction of side population cells, the expression of ABCG2 was correspondingly increased in the cells treated at 1% O_2_ tension, in comparison with the cells cultivated at 20% O_2_ for both cell lines. Since CD44 is considered a putative surface marker for cancer stem/progenitor cells in breast and prostate cancers [19], [22], [48], [49], we analyzed CD44 expressions in these cells as well. Our study showed that CD44 expression was significantly induced under hypoxia. The putative prostate cancer stem-like cell marker CD44 has been associated with prostate cancer stem like feature [46], and has been indicated to play an essential role in the quiescence of hematopoietic stem cells in the osteoblastic niche [50]. The extended G_0_/G_1_ stage and induced CD44 and ABCG2 expressions in our present study may suggest more slow-cycling cancer stem-like cells under hypoxia, which is in line with the study reported by Ishimoto et al [51].

Both CD44 and ABCG2 have been strongly indicated as stem cell markers in previous studies [19], [52], [53]. In the present study, we examined these two factors in the same cell populations, in order to explore whether their responses to hypoxic treatments were related. Using flow cytometry, we found that most of the PC-3 and DU145 cells were CD44 positive, but only a small portion of cells in these two cell lines were ABCG2 positive. The ABCG2 positive cells were mostly CD44^bright^ cells, and hypoxia induced expressions of CD44 and ABCG2 in both cell lines, indicating that ABCG2 expression may be associated with CD44^bright^ cells. Next, we sorted the CD44^bright^ cells and verified that they were primarily strongly positivity for ABCG2. On the contrary, all the CD44^dim^ cells were almost ABCG2 negative. Furthermore, there were higher levels ABCG2 expressions in the hypoxia pretreated CD44^bright^ cells than the CD44^bright^ cells without hypoxia-pretreatment in both cell lines. Collectively, our results suggest a strong association between ABCG2^+^ and CD44^bright^ cells.

In consistent with previous report that both *NANOGP8* mRNA and Nanog protein are enriched in the CD44^bright^ human prostate cancer cells [16], we also found that higher protein expressions of Oct3/4 and Nanog in the CD44^bright^ cells compared to the corresponding CD44^dim^ cells. Moreover, we examined additional stemness features of these cells using colony formation and sphere growth assays. These experiments showed that the CD44^bright^ cells formed more colonies than the CD44^dim^ cells. The sphere growth assay also showed significantly higher sphere formation efficiency for the CD44^bright^ cells, and this finding is supported by the former report that CD44^bright^ prostate cancer cells display stem –like characteristics such as more proliferative, clonogenic, tumorigenic and metastatic than the corresponding CD44^dim^ cells [54]. Furthermore, the colony efficiency of the CD44^bright^ cells was significantly improved following hypoxic pretreatment, whereas the CD44^dim^ cells did not respond to such hypoxic exposure. Since colony formation and sphere formation capabilities are confined to stem cells [46], [55], [56], these results may support the hypothesis that CD44^bright^ cells possess stem-like properties in the prostate cancer cells [54].

In summary, hypoxia enhanced the stem-like properties of the human prostate cancer cell lines PC-3 and DU145. Hypoxic treatment also induced growth capability of CD44 positive cells in these two cell lines, and CD44^bright^ cells possessed greater stem cell-like features, as verified by higher expressions of stemness factors and ABCG2, and significantly higher colony and sphere formation efficiency. Furthermore, the stem-like properties of the CD44^bright^ cells were significantly increased upon hypoxic pretreatment.
